The article "Environmental Healthcare Assessment via Daily-Scale Drought Monitoring" was retracted in 2023. Reasons: unreliable results or conclusions; concerns about the data; concerns about the peer review; concerns about the citations.

# Environmental Healthcare Assessment via Daily-Scale Drought Monitoring

**DOI:** 10.1155/2022/5010760

**Published:** 2022-04-13

**Authors:** Huizhou Yuan, Qiang Huang, Qiongling Lu, Haiyan Yang, Wei Jie Lu

**Affiliations:** ^1^School of Construction and Environmental Engineering, Shenzhen Polytechnic, Shenzhen 518055, China; ^2^Institute of Urban Ecology and Environmental Technology, Shenzhen Polytechnic, Shenzhen 518055, China

## Abstract

Precipitation is the most important factor in determining the drought condition. In addition, the drought condition is also affected by the hydrological process such as evaporation, leakage, runoff, and groundwater. Based on a simple physical model of water income and recession, the effective precipitation index (WAP) can reflect the drought condition in a region on a short time scale. Using a water decline equation to describe the process of preliminary soil moisture, evaporation, runoff, and groundwater, the WAP can be used for the quantitative study of drought. This paper improves the calculation program of WAP with reference to the calculation model of the standardized index. The improved WAP (called SWAP) effectively solves the problem of seasonality in drought. The results showed that SWAP has the ability to capture the drought processes of occurrence, development, peak, and regression in a short time scale, and the SWAP can be used as an effective tool for drought identification, assessment, and prevention.

## 1. Introduction

Drought is a kind of natural disaster characterized by relative shortage of water. It can occur in any season in any region, causing hundreds of millions of losses every year [1, 2]. Drought is considered as the most damaging natural disaster due to its extensive socioeconomic impacts [3, 4]. Such impacts can either be direct (e.g. restrictions on water use or decreasing crop yield) or indirect (e.g. increasing food costs due to decreased crop yield) [5]. Under the background of global warming, severe drought events have occurred more frequently throughout the world in recent years [6]. Therefore, it is essential to understand the drought processes and enhance the drought monitoring ability for disaster prevention and mitigation.

Drought can be generally classified into four categories: meteorological drought, hydrological drought, agricultural drought, and socioeconomic drought [7]. In general, meteorological drought is considered to be the source of other type of drought [8]. With the transmission of water loss in each link of water cycle, meteorological drought gradually develops into agricultural drought, hydrological drought, and economic drought. Due to the complex mechanism of drought, there is no unified and complete definition of drought in the world [9]. According to the meteorological data of the Midwestern United States for several years, Palmer [10] proposed the PDSI (the Palmer index) based on the concept of “climate suitable precipitation for the current situation.” This was the first comprehensive effort to assess the total moisture status of a region. Considering a number of sources of water income and expenditure that affect the drought condition, PDSI has a clear physical meaning. A self-calibrating version of PDSI introduced by Wells et al. [11] is widely used in drought monitoring. However, PDSI is limited to the characteristics of local climate, soil, and vegetation, which reduces its scope of application when it comes to the comparison in different places. SPI is another widely used index proposed by Mckee et al. [12]. Fitted to a gamma or Pearson type III distribution, each monthly precipitation figure is transformed onto a standard normal form. The probabilistic nature of SPI allows it to be spatially comparable, while its ease of calculation makes it more applicable than many other indices [13]. However, SPI has neglected other important factor affected drought condition [14, 15], especially in light of a general temperature increase over the past 150 years [16, 17]. Considering that evapotranspiration is also an indispensable element in the process of regional water conversion, it also plays an important role in the formation and evolution of drought. Vicente-Serrano et al. [15] proposed a standardized precipitation evapotranspiration index (SPEI) based on SPI. Kao and Govindaraju [18] considered the incomparability of the standardized index on the time scale and further proposed the Joint Drought Index (JDI). Recently, studies found that compound abnormal climate conditions can trigger rapid development of drought [19, 20].

The article "Environmental Healthcare Assessment via Daily-Scale Drought Monitoring" was retracted in 2023. Reasons: unreliable results or conclusions; concerns about the data; concerns about the peer review; concerns about the citations.

Although standardization indices have been widely used in drought researches [21–23], there are still deficiencies. Firstly, the probability of occurrence of droughts in different locations is assumed to be the same, so the standardized index cannot identify those places where droughts occur frequently. Secondly, the standardized index cannot be used for short time drought monitoring (such as daily and weekly scales). For example, for a certain day when no precipitation appeared, the water storage would be regarded in dry state monitored by standardized indices. It is because that the zero value of no precipitation is minimum compared with the long-term historical records. But actually, this day would not be in dry condition if precipitation occurred in previous few days. In addition, the short time drought forecast can provide important guidances for water resource management and crop production. In order to overcome the shortage of the standardization index, Lu [24] proposed a daily weighted average precipitation (WAP), using a water income and recession physical model to characterize the current drought and flood conditions based on current and previous precipitation. The WAP is actually a drought index based on the concept of effective precipitation. It has physical meaning and can reflect the drought conditions in a region on short time scales. Like other drought indices, the results of drought monitoring by WAP would be affected by the seasonality and regional difference of precipitation. To solve this problem, we made some revisions of the calculation model of WAP in this study. Calendar month was used as the unit of calculation to eliminate the seasonality of precipitation, and the WAP value was expressed in the form of probability of occurrence similar with the standardized index to improve its spatial comparability. The novelty of our study is that we made a calculation improvement of the WAP to solve the problem of seasonality and spatial comparability in precipitation. The objectives of this study are (1) to make a calculation improvement of WAP, (2) to compare the superiority of modified WAP with the common used drought indices, and (3) to explore the effectiveness and reliability of the modified WAP in drought monitoring on a short time scale.

## 2. Study Area and Dataset

This study applied the Effective Precipitation Index on drought monitoring in Shaoguan area as a case study. The Shaoguan area is located in the northern mountainous area of Guangdong province in China (Figure 1), which is in the junction between coast and inland. Compared with the developed areas of the Pearl River Delta, the Shaoguan region is one of the few poverty-stricken areas in the province and is the main agricultural production base of the province. In addition, Shaoguan is the source area of the Beijiang River, one of the major tributaries of the Pearl River in southern China, which is playing an important role in flood control and water supply for the downstream cities. Affected by the monsoon climate, abundant precipitation is falling down in Shaoguan area but unevenly distributed during the year. As a result, frequent droughts occurred in the region, causing large agriculture failures and water resources crisis [25]. The future warming trend is projected to exceed 1°C decade^−1^ in this region, and extreme weather such as heat wave is expected to increase, possibly leading to more severe drought events [26]. Finding an effective tool to make a comprehensive understanding of drought processes is of great importance for dealing with the potential threats caused by future droughts in this region.

The article "Environmental Healthcare Assessment via Daily-Scale Drought Monitoring" was retracted in 2023. Reasons: unreliable results or conclusions; concerns about the data; concerns about the peer review; concerns about the citations.

A 0.5° × 0.5° grid dataset was collected from the Meteorological Information Center, China Meteorological Administration (http://data.cma.cn/). The dataset is processed by observation data of 2,416 stations and dem data of 0.5° × 0.5° nationwide, which has undergone strict quality control with good representation and integrity. Data from 15 grids covering the Shaoguan area, including daily precipitation and temperature data from 1961 to 2011, were selected for the study.

## 3. Methodology

### 3.1. Weighted Average Precipitation Index (WAP)

Precipitation is the most essential factor in determining the drought and flood processes. Besides, the drought and flood processes can also be affected by the hydrological processes such as evaporation, leakage, runoff, and groundwater. For example, if there was a large amount of precipitation on a certain day, the flood state would be aggravated, but it did not mean that the day was in a state of flood; and if there was no precipitation or little precipitation, the dry state would be aggravated, but the day was not necessarily in a dry state. That is to say, the amount of precipitation on the day was a necessary condition for determining the state of the drought and flood for current day, but not a sufficient condition. The state of drought and flood on the day depended on the reserve status of the previous moisture (soil moisture, vegetation, discharge, groundwater, etc.). Precipitation increased the water storage on the land surface, and after the precipitation, the water storage on the land surface showed a gradual decline. The water storage declined on rainy days was mainly affected by runoff, while the water storage declined on rainless days was mainly affected by evapotranspiration [24]. Since the hydrological process of precipitation, runoff, and evapotranspiration is a slow cyclic process, the storage change of the previous moisture is also a slow decline process, which can be expressed by a simple physical model [24]:

(1) $$\begin{array}{c} \frac{f\left(t\right)}{\text{d}t}=-bf\left(t\right)+P\left(t\right), \end{array}$$

where *f* (*t*) represents the drought and flood state in a region and *t* is the time. Based on (1), the drought and flood state process in a region is controlled by the two parts of income and expenditure for water storage. The precipitation is the part of the water income in the model, and the water expenditure is expressed by the decline of the water storage, which represents the intensity of the recession. After a series of mathematical integrals and transformations for (1), the current drought and flood state of a region can be simplified to be expressed only by precipitation [24]:

(2) $$\begin{array}{c} f_{0}=\sum_{n=0}^{N}a^{n}P_{n}, \end{array}$$

where *a* is the parameter used to control the contribution of previous precipitation to the current drought and flood state of a region and can be expressed as *a*=exp(−*b*Δ*t*) < 1 (Δ*t* is the time interval taken as one day). *P*_*n*_ represents the amount of precipitation from the current number of days (i.e. *P*_0_ represents the amount of precipitation on the day, and *P*_1_ represents the amount of precipitation from the preday). *N* is the total number of days whose water storage affecting the current drought and flood condition. According to (2), the contribution of the previous precipitation to the current drought and flood state is decreasing, with the days increasing. *N* can be determined by the parameter *c* which is a minimum percentage threshold for the contribution of the previous precipitation to the current drought state. Actually, the current drought and flood state is the result of the weighted accumulation of the water storage which is mainly determined by the previous precipitation. So the *f* value calculated by (2) is an absolute value; thus, it is difficult to distinguish the drought grade, which is important in the actual drought monitoring. Setting weighting coefficients, the *f* value in (2) can be converted into a relative value to distinguish the drought grade:

(3) $$\begin{array}{c} \text{WAP}=\frac{\sum_{n=0}^{N}a^{n}P_{n}}{\sum_{n=0}^{N}a^{n}}. \end{array}$$

WAP is the Weighted Average Precipitation Index, also known as the Effective Precipitation Index, which can be calculated according to any scale above the day. The contribution of the previous precipitation to the current state of drought and flood would be considered as the same by taking a fixed value of 1 for the parameter *a*. That is, WAP would be converted into the a average value during the period of interest (like the calculation mode of SPI). Equation (3) can be further simplified as [24]

(4) $$\begin{array}{c} \text{WAP}=\sum_{n=0}^{N}w_{n}P_{n},\\ w_{n}=\left(1-a\right)a^{n}. \end{array}$$

Shaoguan area is located in the humid area of southeast China. The time of water conversion is about two months [27]. So, the value of *N* can be taken as 60 days, *c* taken as 1%, and then the parameter *a* ≈ 0.93. According to the statistics of drought in agriculture production, Shaoguan area suffered severe droughts in 1963 and 2009.  Figure 2 shows the results of drought monitoring by WAP in 1963 and 2009 using the data from Shaoguan station, which represents the point process of drought. It can be clearly seen from Figure 2(a) that the WAP values are below the average level for most of 1963, which means that there would be a drought in 1963 in Shaoguan area. This situation is severe in the late May and early June of the year. From the results of Figure 2(b), the WAP values are also below the average level for the most of 2009, indicating a drought state throughout the year of 2009. From the comparison, the drought in 1963 would be more severe than that of 2009.

The article "Environmental Healthcare Assessment via Daily-Scale Drought Monitoring" was retracted in 2023. Reasons: unreliable results or conclusions; concerns about the data; concerns about the peer review; concerns about the citations.

### 3.2. Modified Weighted Average Precipitation Index

Due to the uneven spatial and temporal distribution of precipitation in the Shaoguan area, there is a large difference in precipitation between different regions and seasons. The regional differences in precipitation make WAP inevitably have limitations in spatial horizontal comparison. Referring to the standardized index calculation model, converting the WAP into a standardized value can effectively solve the problem of poor spatial compatibility of the WAP. Since the traditional calculation model of the standardized index is based on the historical mean of long-range precipitation sequences, the existence of seasonal differences in precipitation makes the precipitation in a certain season always more or less than the historical average, that is, in a wet or dry state. The situation would be prominent in the monsoon climate zone. This is not the same as the actual situation. Kao and Govindaraju [18] proposed a method in which the precipitation sequence would be divided into 12 subsequences based on the month. Then, the calculation procedure of standardized index is applied to each subsequence, and the calculated results of each subsequence would be reordered time by time to form the final sequence. This modified procedure can reduce the influence of the seasonality in precipitation, which would disturb the results of agricultural drought monitoring. The modified WAP would still capture the physical meaning in water cycle.

According to (1)–(3), WAP is a linear combination of precipitation. Based on the hypothesis that precipitation is subject to the Gamma distribution, WAP must also obey the Gamma distribution [28]. The probability of WAP occurrence in the month is calculated by using the Gamma distribution in units of months. The value obtained after standardization is recorded as SWAP, which is the abbreviation of standardized weighted average precipitation index. Each sequence of SWAP is arranged in chronological order to be the SWAP of the entire sequence.

(5) $$\begin{array}{c} \text{SWAP}=\left\{{\text{SWAP}}^{1},{\text{SWAP}}^{2},\ldots ,{\text{SWAP}}^{12}\right\}. \end{array}$$

Figure 3 shows the comparison of the SWAP calculated by the conventional standardized method with the improved SWAP for monitoring the drought in 1963 and 2009 in Shaoguan area. As shown in Figure 3(a), the results of drought monitoring by SWAP calculated by the conventional method does not faithfully reflect the drought state from April to September in 1963 as shown in Figure 2(a), and the improved SWAP accurately captured this drought state. Moreover, the SWAP calculated by the traditional method incorrectly indicates no drought state from late November to December in 1963, but a flood state is shown in Figure 2(a). In contrast, the improved SWAP also accurately reflects the actual situation. Similarly, from the results shown in Figure 3(b), the SWAP calculated by the conventional method fails to monitor the drought condition in May, August, and September of 2009 and the flood condition in December and November shown in Figure 2(b). Conversely, the results of the improved SWAP reflect the actual situation. Therefore, due to the seasonality in precipitation, the SWAP calculated by the traditional standardized method has disadvantages in drought monitoring. The improved SWAP effectively reduces the calculation error caused by the seasonality of precipitation and improves the accuracy for drought monitoring.

The article "Environmental Healthcare Assessment via Daily-Scale Drought Monitoring" was retracted in 2023. Reasons: unreliable results or conclusions; concerns about the data; concerns about the peer review; concerns about the citations.

Following a similar calculation procedure, the SWAP has the same classification of drought levels as the standardized indexes such as SPI, SPEI, and JDI. The traditional standard for drought grade classification is based on the mathematical inflection point of normal distribution curve. Researches show that the drought grades classified by the probability of occurrence (recurrence period) is more suitable in drought monitoring [29, 30]. With the probability of occurrence of 0.3, 0.2, 0.1, 0.05, and 0.02, respectively (recurrence period of 3, 5, 10, 20, and 50 years, respectively), five drought grades can be divided (Table 1).

## 4. Results and Discussions

### 4.1. Correlation with the Standardized Indexes and CI

The Integrated Meteorological Drought Index (CI) is the most commonly used indicator in drought monitoring and assessment for China's government department. CI is a combination of 30 days and 90 days of standardized precipitation index and a relative wetness index of 30 days. Although CI is an empirical index, its results would be authoritative in the current drought monitoring and assessment work in China. Therefore, comparisons would be made between CI and SWAP results to verify the accuracy and effectiveness of SWAP in drought monitoring. The SWAP value would be first transformed to a monthly sequence to make a comparison with the standardized indexes like SPEI and JDI, then the CI. The results are shown in Table 2. SWAP has a high positive correlation with the SPEI, JDI, and CI (Kendall correlation coefficient >0.5), indicating that SWAP shows good consistency with the commonly used drought indexes, thus would be effective in drought monitoring. Besides, the correlation between SWAP and SPEI and JDI and CI is more significant than that of WAP. It also shows that SWAP based on a improved calculation procedure is better than WAP in drought monitoring.

The article "Environmental Healthcare Assessment via Daily-Scale Drought Monitoring" was retracted in 2023. Reasons: unreliable results or conclusions; concerns about the data; concerns about the peer review; concerns about the citations.

### 4.2. Point Process of Drought Monitored by SWAP

SWAP was used to monitor the agricultural drought process in Shaoguan area in 1963 and 2009. The point process of the 1963 and 2009 drought is shown in Figure 4. Compared with the results monitored by WAP shown in Figure 2, the results from SWAP and WAP display a high consistency in drought monitoring, which represents the actual situation. The SWAP results can especially describe the beginning, ending time, duration, severity, and development process of drought. As shown in Figure 4(a), the drought in 1963 began in early April, the early flood season. Five months later, the severity of the drought reached its peak in early June and then quickly reduced because of the sufficient precipitation. A redevelopment process could be found in late July. The drought ended in mid-September and lasted 168 days.

In contrast, the drought in 2009 started in late July, and ended in early November, which lasted 113 days. From Figure 4(b), a three-month development process could be found, after which the severity of the drought reached its peak in late October, then quickly subsided. Comparing the SWAP value of drought period in 1963 and 2009 with those of the same period of the two years before and after, respectively, we found that both the years before and after the drought period were in a flood state. This situation highlights the drought in 1963 and 2009 to a certain degree. Besides, the drought in 1963 was a bimodal type of drought, and the drought in 1963 was a unimodal type of drought. From the perspective of drought severity, the drought in 1963 was more prominent than the 2009 drought in terms of duration and severity.

### 4.3. Spatial Process of Drought Monitored by SWAP

Drought is a natural disaster covering a wide range in space. Accurate monitoring of the spatial process of drought is important for the assessment and prevention of drought. High spatial resolution-gridded data just provides favorable conditions for the monitoring of spatial process of drought. Using the gridded SWAP to monitor the spatial process of drought, we can clearly understand the whole process of drought from development to regression. First, a percentage threshold of 10% is used to determine the beginning and termination time of the drought. That is, if the percentage of grids in which the SWAP value indicates a drought state exceeds the threshold, it is determined that drought begins, and the corresponding time is the beginning time of the drought. Similarly, the termination time of the drought can be determined. Note that drought begins when the percentage of girds in a drought state exceeds the threshold from a lower value and end when the percentage of girds in a drought state less than the threshold from a higher value.

The article "Environmental Healthcare Assessment via Daily-Scale Drought Monitoring" was retracted in 2023. Reasons: unreliable results or conclusions; concerns about the data; concerns about the peer review; concerns about the citations.

Dynamic monitoring of the drought in 1963 in time and space by SWAP is displayed in Figure 5. From the figure, we can see that this drought began in the southern part of the region. The beginning time of the drought can be determined as April 1st. The spatial process of the drought is beginning in southern part, then expanding from the southwest to the northeast. Drought severity was increasing and reached the peak stage in June 6th. From then on, a recession occurred till July 30th, at which the drought develop again. The drought severity was increasing again, and another peak stage occurred in August 31th, with high severity in the whole region. Finally, the drought ended in September 22th. From the results of drought monitoring in time and space by SWAP, the drought in 1963 can be divided into 7 stages: beginning (April 26th), development (May 8st to June 5th), peak (June 6th), recession (June 14th to July 23th), redevelopment (July 24th to August 30th), repeak (August 31th), and end (September 22th). To verify the accuracy of drought monitoring by SWAP, the results of SWAP are compared to those of JDI, which are shown in Figure 6. The monitoring results are consistent from the occurrence of drought to the peak stage. However, due to the limitation of JDI in calculation procedure, JDI can only monitor drought on a month scale. As seen in Figure 6, the results of JDI can not reflect the drought process in detail, which represent the average severity of the whole month. Therefore, it is impossible to understand from the monitoring results of JDI that the drought in 1963 had experienced two peak development processes, and it is impossible to know the exact time of beginning and end. Furthermore, deviations were found in drought monitoring by JDI. From the results of JDI, drought severity in June was less than that in July, but according to the results of SWAP, the drought was in a peak stage in June 6th with the highest severity across the drought period. Another deviation in drought monitoring by JDI is the result in August, which indicate a severe drought. But from the results of SWAP, another peak stage occurred in August 31th, which meant that the drought severity in August 31th was the highest one in the whole August. Obviously, this result was not consistent with that of JDI, that is, the result of JDI in August failed to monitor the actual drought. Besides, the monitoring results of JDI can not show a bimodal process across the drought period. Therefore, the daily-scale SWAP is superior to the monthly-scale JDI in drought monitoring, including detecting the beginning time, end time, and drought development process.

The article "Environmental Healthcare Assessment via Daily-Scale Drought Monitoring" was retracted in 2023. Reasons: unreliable results or conclusions; concerns about the data; concerns about the peer review; concerns about the citations.

Dynamic monitoring of the drought in 2009 in time and space by SWAP is displayed in Figure 7. This drought began in the southern part of the region like the drought 1963 and expanded to the northern part in the development stage. Unlike the drought in 1963, this drought was a type of unimodal drought, which experienced a process of beginning-development-peak-end. So, 4 stages can be divided in this drought: beginning (July 22th), development (July 26th to October 28th), peak (October 29th), and recession (November 12th), lasting 113 days. As seen in Figure 8, the JDI monitoring results also failed to detect the development process and recession process of this drought.

### 4.4. Discussion

Based on a simple physical model to describe regional water income and recession, the Weighted Average Precipitation Index used a modified calculation procedure developed to monitor the drought processes in 1963 and 2009 in Shaoguan area, southeast of China. This drought index called SWAP is based on the concept of effective precipitation, which can better model the previous water storage, including soil moisture, evapotranspiration, discharge, and groundwater. These hydrological processes play an essential role in the formation and development of droughts. The SWAP thus can quantitatively characterize droughts on a short time scale.

The purpose of using a modified calculation procedure to calculate SWAP is to reduce the influence of seasonality in precipitation and improve its spatial comparability. Results showed that the SWAP calculated by the modified procedure is superior to that calculated by the traditional method in drought monitoring. That is, the SWAP calculated by the modified procedure improves the accuracy of drought monitoring. Besides, SWAP showed a high consistency with the commonly used drought indices such as Standardized Index (SI) and Integrated Meteorological Drought Index (CI), which proved the effectiveness of SWAP in drought monitoring.

For the two severe droughts recorded in the Shaoguan area of history, the SWAP performed well in monitoring their development in both time and space. These two droughts belong to two different types of drought. The drought in 1963 was a type of bimodal drought, which experienced a process of beginning-development-peak-recession-redevelopment-repeak-termination. The drought in 2009 was a type of unimodal drought, which experienced a process of beginning-development-peak-termination. To verify the advantage of SWAP in drought monitoring, the results of JDI were used to make a comparison. Results of the comparison showed that the daily-scale SWAP is superior to the monthly-scale JDI in drought monitoring, including detecting the beginning time, termination time, and drought development process.

The article "Environmental Healthcare Assessment via Daily-Scale Drought Monitoring" was retracted in 2023. Reasons: unreliable results or conclusions; concerns about the data; concerns about the peer review; concerns about the citations.

There are some limitations needed to improve in future studies. Firstly, the length of data used to calculate the SWAP in this study should be extended to further investigate the long-term drought processes. Secondly, the SWAP needed to be applied in different climate zone to prove its extensive applicability in drought monitoring.

## 5. Conclusions

1. Based on the concept of effective precipitation, the drought or flood state of certain region depends on both the current and previous water storage. The drought index WAP has a physical meaning of water income and recession, which can be used to quantitative research on droughts.
2. Following a similar calculation model of standardized indexes, a daily-scale drought index SWAP can be developed. Using a modified calculation procedure to reduce the influence of the seasonality of precipitation, the accuracy and effectiveness of SWAP in drought monitoring improves.
3. SWAP provides a clear picture of the drought processes in both time and space, including the beginning time, termination time, and development process of droughts, providing an effective tool for drought identification, assessment, and prevention.

## Figures and Tables

**Figure 1:** Locations of the Shaoguan area with major rivers and grids.

**Figure 2:** The point process of the 1963 and 2009 drought monitored by WAP.

**Figure 3:** Comparison between the SWAP calculated by conventional method and modified method.

**Figure 4:** The point process of the 1963 and 2009 drought monitored by SWAP.

**Figure 5:** The spatial process of the 1963 drought monitored by SWAP including 7 stages: (a) beginning (April 26th), (b) development (May 8st to June 5th), (c) peak (June 6th), (d) recession (June 14th to July 23th), (e) redevelopment (July 24th to August 30th), (f) repeak (August 31th), and (g) end (September 22th).

**Figure 6:** The spatial process of the 1963 drought monitored by JDI.

**Figure 7:** The spatial process of the 2009 drought monitored by SWAP including 4 stages: (a) beginning (July 22th), (b) development (July 26th to October 28th), (c) peak(October 29th), and (d) end (November 12th).

The article "Environmental Healthcare Assessment via Daily-Scale Drought Monitoring" was retracted in 2023. Reasons: unreliable results or conclusions; concerns about the data; concerns about the peer review; concerns about the citations.

**Figure 8:** The spatial process of the 2009 drought monitored by JDI.

**Table 1:** Categories of drought grade for the SWAP.

SWAP value	Probability of occurrence	Drought condition
(−0.84, −0.52]	(0.20, 0.30]	Mild drought
(−1.28, −0.84]	(0.10, 0.20]	Moderate drought
(−1.64, −1.28]	(0.05, 0.10]	Severe drought
(−2.05, −1.64]	(0.02, 0.05]	Extreme drought
<−2.05	<0.02	Exceptional drought

**Table 2:** Correlation between the WAP and SWAP and SPEI, JDI, and CI.

Kendall correlation coefficient	SPEI	JDI	CI
WAP	0.32	0.31	0.57
SWAP	0.61	0.52	0.62

## Data Availability

The data used in this study, a 0.5° × 0.5° grid dataset, were collected from the Meteorological Information Center, China Meteorological Administration (http://data.cma.cn/).

## Additional Points

*Highlights*. (1) We modify the calculation method of WAP to enhance its accuracy for drought monitoring. (2) The modified version of WAP called SWAP was used to reanalyze the drought processes in Shaoguan area, China, on a daily scale. (3) The SWAP provides a clear picture of the drought processes in both time and space.
